# A Report of 61 Cases of Retroperitoneal Laparoscopic Nephron-Sparing Surgery and Factors Affecting Postoperative Renal Function

This article has been retracted.

**DOI:** 10.1155/2021/2283727

**Published:** 2021-10-16

**Authors:** Yao Song, Songqiang Pang, Jinqiang Yang, Sen Li, Yaqiang He, Gongtang Luo

**Affiliations:** Department of Urology, Shunyi Hospital, No. 3, Guangming South Street, Shunyi District, Beijing 101300, China

## Abstract

**Objective:**

To explore the situation of 61 patients with renal tumors who underwent retroperitoneal laparoscopic nephron-sparing surgery (RLNSS) and the factors affecting postoperative renal function.

**Methods:**

A total of 61 patients with renal tumors who underwent RLNSS in our hospital from January 2018 to January 2021 were included in this study. All patients were treated with RLNSS. The clinical data of patients were recorded. Before operation and 3 months after operation, the change value of glomerular filtration rate (ΔGFR) was measured by the Gates method. Multivariate linear regression was used to analyze the related factors affecting postoperative renal function.

**Results:**

All 61 patients successfully completed the operation. The mean operative time was 60–150 min‚ average (98.75 ± 14.38) min. The estimated intraoperative blood loss was 20–310 ml‚ average (107.93 ± 68.55) ml. Intraoperative warm ischemia time (WIT) was 0–39 min, with an average of (21.16 ± 6.47) min. All patients' pathological margins were negative after operation. In all patients, there were 5 postoperative complications, including 2 cases of renal wound bleeding (3.28%), 1 case of hematuria (1.64%), 1 case of urinary fistula (1.64%), and 1 case of subcutaneous emphysema (1.64%). There were significant differences in tumor diameter, preoperative GFR, operation time and WIT (*P* < 0.05). Multivariate analysis showed that tumor diameter, preoperative GFR, and WIT were all factors affecting the postoperative renal function of patients with RLNSS (*P* < 0.05).

**Conclusion:**

RLNSS has a good curative effect on patients with renal tumor, and tumor diameter, preoperative GFR, and WIT were all factors affecting the postoperative renal function of patients with RLNSS.

## 1. Introduction

9Renal tumors are frequent urinary system tumors in clinic, which are mainly caused by heredity, environment, obesity, smoking, hypertension, and other causes, and patients are mainly accompanied by clinical symptoms such as lumbago, hematuria, lumps, and other symptoms [1]. It has been reported that the incidence of renal tumors ranks second in urinary system tumors, second only to bladder tumors, and accounts for about 2%-3% of adult malignant tumors. Renal tumors are more common in people aged 50–70 years, and males are higher than females, among which malignant tumors account for about 95%, while benign tumors are rare, and the prevalence rate is gradually increasing in recent years, causing great harm to the life safety of patients [2]. Therefore, it is of great significance to take effective measures to treat patients with renal tumors.

At present, with the continuous development of medical imaging technology, the detection rate of early renal cancer is increasing. At the same time, the continuous improvement of surgical techniques also provides technical support for nephron-sparing surgery for patients with renal tumors. Laparoscopic nephron-sparing surgery (LNSS) was first applied to animal experiments by the team of scholar McDougal in 1993 [3]. Winfield's team implemented the first clinical LNSS in 1993 [4]. In recent years, with the continuous improvement of medical technology and operation level, retroperitoneal laparoscopic nephron sparing surgery (RLNSS) is the main treatment for renal tumors. RLNSS adopts the posterior approach to completely remove the renal tumor tissue, which can completely remove the tumor while preserving the residual nephron and function of the affected renal as much as possible. RLNSS has the characteristics of being safe and effective, short operation time, small damage, and rapid recovery. The mortality, recurrence rate, and tumor-free survival rate of RLNSS are comparable to those of radical nephrectomy [5, 6].

However, although the renal function of most patients with renal tumors recovered well after RLNSS, some scholars found that the renal function of some patients with renal tumors recovered poorly after RLNSS. Ebbing's team [7] reported that the incidence of renal failure and cardiovascular events in patients with renal tumors after LNSS is low, but renal failure may occur, and the influence of different surgical conditions on postoperative renal function decline is still controversial. Therefore, it is particularly important to observe and analyze the influencing factors of renal function in patients with renal tumors after RLNSS. At present, there are many clinical evaluation indexes about renal function after RLNSS operation, among which the glomerular filtration rate (GFR) for evaluating glomerular filtration function refers to the amount of ultrafiltrate produced by the two renals per unit time, which is not only a common serological index reflecting the renals' drainage and detoxification ability but also an important reference index for diagnosis, staging, and drug use of renal diseases [8].

Our doctor observed 61 patients with renal tumor undergoing RLNSS and analyzed the factors affecting renal function after RLNSS, in order to ensure good operation effect and improve the renal function of patients and provide theoretical reference for the optimization of clinical medical work.

## 2. Materials and Methods

### 2.1. Research Object

A total of 61 patients with renal tumors who underwent RLNSS in our hospital from January 2018 to January 2021 were included in this study. Among them, there were 39 males and 22 females, aged 39–75 years, with an average age of (56.01 ± 13.26) years and a course of 1 month to 9 years. 32 patients were found by routine physical examination or other systemic diseases, 21 patients were unwell due to soreness of the waist, and 8 patients were hospitalized due to gross hematuria, persistent low fever, and abdominal mass. All patients were examined by abdominal ultrasound, abdominal CT, renal CTA, intravenous urography, chest radiograph, or lung CT before operation, so as to make clear the renal occupation. 42 cases of renal cell carcinoma were diagnosed before operation, including 22 cases of T1aN0M0, 18 cases of T1bN0M0, and 2 cases of T2aN0M0; there were 19 cases of renal hamartoma. The tumor was 1.3–6.0 cm in diameter, with an average diameter of (3.73 ± 1.02) cm. Tumor lesion site: 41 cases on the left side and 20 cases on the right side. There were 43 cases with tumor protruding from the surface and 18 cases with tumor located on the surface of the renal but not protruding from the surface of the renal. Tumor location: 12 cases were located in the upper pole of the kidney, 23 cases in the kidney in central, and 26 cases in the inferior pole of the kidney.

Inclusion criteria: ① No tumor thrombus in the renal vein and vena cava was found in imaging examination, and no distant metastasis such as lymph nodes, liver, and lung was found. ② Routine blood tests, blood biochemistry, and other indexes were performed on patients, and all patients were planned to undergo RLNSS operation, and all patients had no contraindications. ③ All patients were performed RLNSS by the same operator.

Exclusion criteria: ① Patients had contraindications of general anesthesia and chronic renal diseases such as chronic glomerular diseases. ② The patient was complicated with ureteral calculi and hydronephrosis. ③ Congenital anatomical malformation of the urinary system, such as duplicate renal, duplicate ureter, and horseshoe renal.

### 2.2. Methods

1. Operation: all patients were given general anesthesia plus endotracheal intubation. They took the healthy lateral position and raised the lumbar bridge. After preparing the conventional abdominal operation space and placing the cannula with three holes, a long incision of 3 cm was made with a sharp knife in front of the psoas major muscle 2 cm below the 12th costal margin of the posterior axillary line. After the greater curvature was bluntly separated to the retroperitoneum, and a visual balloon dilator was inserted to inflate the retroperitoneal space. Under the guidance of the index finger, 10 mm and 5 mm Trocar were placed in the anterior axillary line 2 cm above the iliac crest and under the rib, respectively, and the cannula was retained, while the 12 mm Trocar cannula was retained in the posterior axillary line. The laparoscope was placed into the retroperitoneal space, and the fat tissue outside the peritoneum and Gerota fascia was sharply separated to the iliac fossa by using an ultrasonic scalpel, which enlarged the retroperitoneal cavity and fully exposed the retroperitoneal structure. We carefully identified the retroperitoneal fold and cut the Gerota fascia longitudinally. We freed perirenal fat as close to the tumor as possible to fully expose the renal tumor. If it could be definitely hamartoma with large volume, it was not necessary to completely free the tumor to avoid obvious bleeding. We looked for the free renal artery outside the perirenal fat sac and blocked the renal artery with a bulldog clamp. Infusion of inosine 1 g before renal artery occlusion was carried out. Also, a “J”-shaped electric hook or ultrasonic knife was used to cauterize a circle 0.5 cm away from the tumor edge (Hamartosis Nephroma <0.5 cm) to mark the tumor resection range. After the renal artery was blocked, the tumor and its surrounding tissues were quickly excised with scissors along the marking line, and some bleeding places were stopped with automatic ligation forceps. The operation was performed along the outside of the tumor capsule to prevent damage to the capsule and carefully observe the wound surface of the renal to ensure that there was no residual tissue. After the tumor was completely removed, if the collecting system was found to be damaged during the operation, the collecting system should be sutured with 3-0 absorbable suture first, then the renal parenchyma wound should be sutured with 1-0 absorbable suture, and the knot should be replaced by automatic ligating forceps intermittently. The bulldog clamp was released to restore renal blood supply and reduce pneumoperitoneum pressure to about 0.5 kPa. After there was no active bleeding observed, a hemostatic gauze was used to cover the suture. The specimen was put into a specimen bag and taken out. The drainage tube was placed around the renal, and the incision was closed.
2. The clinical data of all patients were recorded, including age, gender, hypertension, diabetes, tumor location, tumor diameter, pathological type, preoperative GFR, operative time, intraoperative blood loss, and warm ischemia time (WIT).
3. Before and 3 months after operation, GFR was measured by the Gates method, GFR of both the renals was measured by SPECT renal dynamic imaging, and GFR changes (ΔGFR) before and after operation were recorded. Medical staff told patients to drink about 300–500 ml of water and empty their bladder 20 min before examination. Imaging agent (99mTc-DTPA, 1 mL) was shot injected into the elbow vein, and then, SPECT was used to scan immediately. The blood phase was 2s/frame for 1 min, and the functional phase was 60 s/frame for 25 min, and images were collected. The contour of the renal was outlined by region of interest (ROI) technology, and the crescent background area was outlined at the lower edge of the renal. The computer software automatically generates the time-radioactivity curve of the renal, and the GFR of the renal was obtained.

### 2.3. Statistical Methods

SPSS22.0 software was used for statistical analysis. The measurement data were in accordance with normal distribution, and the *t*-test and variance test were used to compare the measurement data. Multivariate linear regression was used to analyze the factors affecting postoperative renal function. *P* < 0.05 was the difference with statistical significance.

## 3. Results

### 3.1. Operation Conditions

All 61 patients successfully completed the operation, no death occurred during the operation, and no patients were converted to laparotomy during the operation. The mean operative time was 60–150 min‚ average (98.75 ± 14.38) min. The estimated intraoperative blood loss was 20–310 ml‚ average (107.93 ± 68.55) ml. The mean GFR value of diseased kidney preoperative was (43.32 ± 11.96) ml/min, the GFR value of nondiseased kidney preoperative was (34.85 ± 12.70) ml/min, and the mean GFR value of diseased kidney postoperative was (29.17 ± 13.22) ml/min. Intraoperative WIT was 0–39 min, with an average of (21.16 ± 6.47) min. Among them, there were 2 cases with 0 ischemia time: 1 case had the largest tumor diameter of 1.5 cm, and the tumor was located at the upper pole of the kidney. CT showed that the tumor was superficial, and according to the intraoperative situation, the renal artery was not blocked; in another patient, the largest tumor diameter was 3.2 cm, and the tumor was located at the inferior pole of the kidney. CT showed exogenous growth, and according to the intraoperative situation, the renal artery was not blocked.

### 3.2. Postoperative Pathological Results

All patients' pathological margins were negative after operation. Postoperative pathology confirmed 20 cases of renal hamartoma, 37 cases of clear cell carcinoma, and 4 cases of renal papillary adenocarcinoma. The postoperative retroperitoneal drainage tube was indwelled for 7–10 days, and the urethral catheter was indwelled for 5–9 days. All patients were cured and discharged and were hospitalized for 10–17 days after operation, with an average hospital stay of (13.8 ± 1.04) days.

### 3.3. Postoperative Complications

In all patients, there were 5 postoperative complications, including 2 cases of renal wound bleeding (3.28%), 1 case of hematuria (1.64%), 1 case of urinary fistula (1.64%), and 1 case of subcutaneous emphysema (1.64%). After active postoperative treatment, all the complications were relieved and no serious complications were found. All patients were followed up for 3–6 months, and all patients survived without tumor.

### 3.4. Univariate Analysis of Influencing Postoperative Renal Function of RLNSS Patients

Age, gender, hypertension, diabetes, tumor location, pathological type, and intraoperative blood loss had no significant effect on the postoperative renal function of patients with RLNSS (*P* > 0.05). There were significant differences in tumor diameter, preoperative GFR, operation time, and WIT (*P* < 0.05). It is displayed in Figure 1.

### 3.5. Multivariate Analysis of Influencing the Postoperative Renal Function of RLNSS Patients

Taking ΔGFR as the dependent variable and taking the tumor diameter, preoperative GFR, operation time, and WIT, which are different in univariate analysis, as independent variables, the multiple linear regression analysis was carried out. Multivariate analysis showed that tumor diameter, preoperative GFR, and WIT were all factors affecting the postoperative renal function of patients with RLNSS (*P* < 0.05). It is displayed in Table 1.

## 4. Discussion

At present, the morbidity and mortality of renal tumors are increasing year by year, which makes the treatment of renal tumors more and more concerned by surgeons. The treatment methods of renal tumors mainly include LNSS, radical nephrectomy, renal artery embolization, and minimally invasive treatment [9]. With the continuous development of medical technology and the continuous progress of imaging, laparoscopic technology has been developed more widely in LNSS. RLNSS is a treatment method that can preserve the renal function of patients to the maximum extent on the premise of resection of renal tumors and has become a common treatment method for renal tumors. Liu's team [10] performed RLNSS on 41 patients with large renal angiomyolipoma, and 35 patients were successfully operated. The median operation time was 167 min, the median WIT was 21 min, the median estimated blood loss was 200 ml, and the median postoperative hospital stay was 6.5 d. The results showed that RLNSS was a safe, feasible, effective, and minimally invasive operation. Compared with open surgery, RLNSS not only has the advantages of fast postoperative recovery and short hospital stay but also is particularly suitable for tumors on the dorsal and lateral back of renal [11]. It has been reported by scholars that the operation time, blood loss, renal ischemia time, hospital stay, incidence of complications, and the amount of postoperative anesthetics in the retroperitoneal route group are superior to those in the intraperitoneal route group [12]. Because of the magnifying effect of laparoscopy, it can ensure clear visual field during operation. Therefore, RLNSS is easy to be accepted by patients because of its advantages of safety, feasibility, less surgical trauma, clear anatomical level, high surgical accuracy, and great safety [13].

In this study, all 61 patients successfully completed the operation, the average operation time was (98.75 ± 14.38) min, and all patients had negative pathological margins after operation. Complete tumor resection and keeping the pathological margin negative are the successful indicators of RLNSS surgery. The range of tumor resection is 0.5 cm away from the normal renal tissue at the margin of the tumor, which can not only effectively retain more nephrons but also ensure the margin negative and reduce the risk of local tumor recurrence. The average estimated intraoperative blood loss was (107.93 ± 68.55) ml. Renal arteriography can help clearly understand the location of the tumor and blood vessel, the anatomy of the blood vessel in the renal, and the blood supply source of the tumor. It is necessary to cut off some blood vessels before operation to reduce the amount of bleeding. In the clinical operation of RLNSS, renal pedicle occlusion is divided into the warm ischemia method and cold ischemia method; the warm ischemia method is to block the renal pedicle at normal temperature, and the cold ischemia method is to block the renal pedicle while supplementing with ice water and ice packs to reduce the kidney temperature [14]. We performed RLNSS operation with warm ischemia, blocked renal artery with a bulldog clamp, and the wound had clear visual field, and inosine was dripped quickly, which was beneficial to protect renal function. When the ischemia time of the renal artery is blocked for more than 30 min, the renal function of patients may be irreversibly damaged, so WIT should be controlled within 30 min, and the average WIT during operation in this study was (21.16 ± 6.47) min. In recent years, due to the strict selection of cases, the improvement of surgical skills, and the accumulation of perioperative experience, the complications of patients with renal tumors undergoing RLNSS have been significantly reduced. We found 5 postoperative complications, including 2 cases of renal wound bleeding, 1 case of hematuria, 1 case of urinary fistula, and 1 case of subcutaneous emphysema. Renal wound bleeding is a common complication after RLNSS operation. It is very important to have a reliable renal parenchyma hemostasis technique during operation to prevent renal wound bleeding. Endoluminal cutting tools, such as bipolar electrocoagulation, ultrasonic scalpel, microwave scalpel, and radiofrequency ablation, have been widely used in RLNSS surgery, which can achieve a satisfactory hemostatic effect. Urinary fistula, as a common complication of RLNSS surgery, can be effectively improved by conservative treatment and urinary catheter and double *J* tube drainage [15]. If the patient has hematuria, it should be based on the patient's degree of hematuria, according to the doctor's advice to take reasonable treatment drugs. If the patient has subcutaneous emphysema, the patient can be cured by giving low-flow continuous oxygen inhalation.

Multivariate analysis showed that tumor diameter, preoperative GFR, and WIT were all factors affecting the postoperative renal function of patients with RLNSS. According to the selection criteria of tumor size for RLNSS surgery, the best index is that the tumor diameter is ≤ 4 cm. However, in the case of solitary renal and double renal cell carcinoma, even if the tumor is > 4 cm, RLNSS can be selected. However, when the tumor diameter is larger than 4 cm, it is difficult to resect the tumor intracavitary, and the suture technique and proficiency under a microscope are required. RLNSS surgery has certain difficulties and risks, which are prone to various complications and seriously affect the quality of life of patients. We found that, with the increasing diameter of renal tumor, the change of GFR value became larger, and the GFR value of the affected renal decreased more after operation. The possible reason is that the larger the diameter of the renal tumor, the less the nephrons can be retained after the complete resection of the renal tumor, and the larger the diameter of the tumor also increases the difficulty of the operation, resulting in prolonged resection and suture time and WIT, which in turn leads to poor renal function after the operation [16]. Patients with low GFR before operation can cause a series of biochemical changes such as decreased renal blood flow, damaged renal blood vessels, and decreased glomerular ultrafiltration coefficient after undergoing renal artery occlusion and tumor resection during RLNSS operation, resulting in decreased ATP, increased oxygen free radicals, calcium overload, and apoptosis in patients' bodies, further leading to pathological changes in the renal parenchyma structure, which will aggravate renal function damage after operation [17]. Therefore, aiming at the patients with low GFR value before operation, the medical staff should make good preparations before operation and take measures to protect the renal function during operation and try their best to reduce the damage of renal function after operation by selecting drugs with less renal toxicity during the perioperative period, actively regulating blood pressure and blood sugar, dropping inosine before renal artery occlusion, and shortening WIT. In addition, we believe that the longer the WIT, the greater the degree of nephron necrosis and the greater the ΔGFR, which will lead to the more serious renal function injury after operation. Irreversible diffusion disorder may occur in the operation renal, and this level will not be decreased. This may be related to the mechanism of renal hypoxia and reperfusion injury. The hypoxic injury of blocking renal blood flow reduces ATP production, destroys the cytosolic membrane structure, causes damage and change of cell membrane structure and permeability, increases the influx of extracellular Ca^2+^, and then, leads to intracellular calcium overload. The increase of intracellular free Ca^2+^ can hinder mitochondrial oxidative phosphorylation, which in turn leads to the decrease of ATP production and cell death [18]. We have carried out RLNSS surgery for many years, and through the inquiry of the literature and our own operating experience, we believe that WIT may be shortened by the following methods: ① Combined with CTA examination, it is necessary to confirm the existence of accessory renal artery, and its position, shape, and branches were determined. ② The blocking is selectively removed sequentially, and it cooperated with the application of ultrasound during the operation. ③ After the renal artery was blocked, the tumor was removed along the labeled line by “scissors cold incision.” ④ We improved the automatic ligation forceps and standardized the suture operations such as stitch distance and depth of stitches. ⑤ No blocking technology was used.

## 5. Conclusions

To sum up, RLNSS has a good curative effect on patients with renal tumor, and tumor diameter, preoperative GFR, and WIT were all factors affecting the postoperative renal function of patients with RLNSS. In this study, 61 patients with renal tumors who underwent RLNSS were satisfied with the short-term curative effect, but the long-term curative effect needed long-term follow-up observation, and there was a limitation that the statistical sample size was not large enough. With the extensive application of endoscopy, it is expected that the influencing factors of renal function after RLNSS can be further confirmed by the analysis of large sample data.

## Figures and Tables

**Figure 1:** Univariate analysis of influencing the postoperative renal function of RLNSS patients.

**Table 1:** Multivariate analysis of influencing the postoperative renal function of RLNSS patients.

Variable	*B* value	*SE* value	*Walds* value	*OR* value	95% CI	*P* value
Tumor diameter	0.447	0.203	4.848	1.563	1.050–2.327	0.021
Preoperative GFR	0.346	0.170	4.142	1.413	1.019–1.972	0.045
Operation time	0.194	0.116	2.796	1.214	0.967–1.524	0.067
WIT	0.382	0.178	4.605	1.465	1.033–2.076	0.033

## Data Availability

The data used and/or analyzed during the current study are available from the corresponding author.

## References

[1] Gray R. E., Harris G. T. (2019). Renal cell carcinoma: diagnosis and management. *American Family Physician*.

[2] Rossi S. H., Klatte T., Usher-Smith J., Stewart G. D. (2018). Epidemiology and screening for renal cancer. *World Journal of Urology*.

[3] McDougall E. M., Clayman R. V., Chandhoke P. S. (1993). Laparoscopic partial nephrectomy in the pig model. *The Journal of Urology*.

[4] Winfield H. N., Donovan J. F., Godet A. S., Clayman R. V. (1993). Laparoscopic partial nephrectomy: initial case report for benign disease. *Journal of Endourology*.

[5] Hoshii T., Morita S., Ikeda Y., Hasegawa G., Nishiyama T. (2017). Laparoscopic retroperitoneal nephron-sparing surgery without renal artery clamping with preoperative selective arterial embolization for management of right renal angiomyolipoma of diameter 10 cm: a case report. *Journal of Endourology Case Reports*.

[6] Li T. T., Feng J., Li Y. L., Sun Q. (2021). A retrospective study of open and endoscopic nephron sparing surgery in the treatment of complex renal tumors. *Pakistan Journal of Medical Sciences*.

[7] Ebbing J., Menzel F., Frumento P. (2019). Outcome of kidney function after ischaemic and zero-ischaemic laparoscopic and open nephron-sparing surgery for renal cell cancer. *BMC Nephrology*.

[8] Zhou Y., Jiang S. M., Li L. (2020). Efficacy and safety of tanshinone for chronic kidney disease: a meta-analysis. *Evidence-Based Complementary and Alternative Medicine: eCAM*.

[9] Escudier B., Porta C., Schmidinger M. (2019). Renal cell carcinoma: ESMO Clinical Practice Guidelines for diagnosis, treatment and follow-up. *Annals of Oncology*.

[10] Liu X., Ma X., Liu Q. (2018). Retroperitoneal laparoscopic nephron sparing surgery for large renal angiomyolipoma: our technique and experience. A case series of 41 patients. *International Journal of Surgery*.

[11] Porpiglia F., Fiori C., Terrone C., Bollito E., Fontana D., Scarpa R. M. (2005). Assessment of surgical margins in renal cell carcinoma after nephron sparing: a comparative study. *The Journal of Urology*.

[12] Mittakanti H. R., Heulitt G., Li H.-F., Porter J. R. (2020). Transperitoneal vs. retroperitoneal robotic partial nephrectomy: a matched-paired analysis. *World Journal of Urology*.

[13] Yang F., Liu S., Mou L., Wu L., Li X., Xing N. (2019). Application of intraoperative ultrasonography in retroperitoneal laparoscopic partial nephrectomy: a single-center experience of recent 199 cases. *Endoscopic Ultrasound*.

[14] Bertolo R., Garisto J., Dagenais J. (2018). Cold versus warm ischemia robot-assisted partial nephrectomy: comparison of functional outcomes in propensity-score matched “at risk” patients. *Journal of Endourology*.

[15] Ye Y.-L., Liang H.-T., Tan L. (2019). Conservative treatment for urinary fistula following ileal conduit urinary diversion: a simple method. *BMC Urology*.

[16] Lin L., Li X., Guan H. (2019). Renal function, complications, and outcomes of a reduction in tumor size after transarterial embolization for renal angiomyolipomas: a meta-analysis. *Journal of International Medical Research*.

[17] Liu J., Tian C., Zhang Z. (2020). Correlation between preoperatively predicted and postoperatively observed renal function using an imaging‑based approach: a retrospective cohort study. *Oncology Letters*.

[18] Rosen D. C., Kannappan M., Paulucci D. J. (2018). Reevaluating warm ischemia time as a predictor of renal function outcomes after robotic partial nephrectomy. *Urology*.

